This article has been retracted.

# Exploration of the Curative Effect of Early Enteral Nutrition Nursing on Patients with Severe Acute Pancreatitis and the Improvement of Patients' Mental Health and Inflammation Level

**DOI:** 10.1155/2021/8784905

**Published:** 2021-09-11

**Authors:** Qigui Xiao, Lan Lang, Zhenhua Ma, Yulin Zhang, Kedong Xu

**Affiliations:** Department of Hepatobiliary Surgery, The First Affiliated Hospital of Xi'an Jiaotong University, Xi'an 710061, Shaanxi Province, China

## Abstract

In order to explore the curative effect of early enteral nutrition nursing on patients with severe acute pancreatitis and the improvement of patients' mental health and inflammation levels, this paper compares the curative effect of early enteral nutrition nursing and traditional care on patients with severe acute pancreatitis and the improvement effects of patients' mental health and inflammation levels through controlled trials. Moreover, this paper combines statistical methods for data processing and visually expresses data through statistical graphs and statistical tables. Through the comparison of experiments, it can be seen that the improvement effect in all aspects of patients in the test group is significantly higher than that in the control group. Finally, through the analysis of the test results, it can be known that the use of early enteral nutrition nursing for patients with acute severe acute pancreatitis has a certain effect in improving their nutritional status, regulating immune function, and promoting mental health.

## 1. Introduction

Severe acute pancreatitis (SAP) refers to the inflammatory reaction of pancreatic tissue self-digestion, edema, hemorrhage, and even necrosis caused by the activation of pancreatin in the pancreas due to various inducements. It is one of the most common clinical acute and critical illnesses, and its main clinical manifestations are abdominal pain, fever, nausea, and vomiting [1]. With the development of the social economy and the improvement of people's living standards, especially high-fat diet and excessive drinking, the incidence of SAP is increasing year by year in the world [2]. SAP has the characteristics of rapid onset, critical illness, and long course of illness. Therefore, patients are prone to negative emotions such as anxiety and depression, which affect the implementation of treatment and nursing measures. Currently, the main place to treat SAP patients is the Intensive Care Unit (ICU). Due to the special ICU environment (no light changes, no family accompany, closed space, equipment alarms, and other noises), patients staying in the ICU are likely to suffer from negative emotions while enduring physical discomfort. Previous studies have shown that different negative emotions in patients can cause excessive tension in the cerebral cortex of patients, leading to endocrine, autonomic, and nervous system dysfunctions, reducing the body's immunity and worsening the disease, triggering a vicious circle [3]. A survey of Bolosi, a foreign scholar, found that patients will undergo a series of psychological disorders after being admitted to the ICU. Among them, more than 80% of patients will have negative emotions such as anxiety/depression. The existence of psychological barriers is not conducive to the recovery of the disease. On the contrary, it will aggravate the condition, prolong the patient's hospitalization time, increase the family's financial burden, and cause a waste of medical resources.

In the 1980s, in the United States, faced with unreasonable growth in medical expenses and problems caused by medical quality and cost, health economists began to study clinical pathways (CPs). The clinical path is an optimized, simplified, and efficient management for the disordered state of patient management. It is the most appropriate treatment and care plan formulated by a group of medical staff to treat and care a certain disease. Moreover, it is an emerging standardized medical management model that can reduce the average hospitalization time and hospitalization cost of a single disease and achieve the expected therapeutic effect. In addition, it is to take an effective approach for a certain disease or operation to achieve the purpose of improving patient services and effectively using health resources. The clinical pathway was originally a method of industrial production engineering management. In 1985, the New England Medical Center in the United States took the lead in implementing the clinical pathway. It proved that the clinical pathway can successfully reduce the high cost in the health system.

There is no report on the incidence of acute pancreatitis in our country. However, in recent years, with the improvement of people's living standards and the change of dietary structure, some small-scale literature reports that the incidence of acute pancreatitis in our country is increasing year by year. The cause of acute pancreatitis varies greatly between regions. Based on reports from various countries, the main causes of acute pancreatitis are still biliary tract diseases and alcohol. The common acute pancreatitis in our country is biliary and hyperlipidemia, closely related to unhealthy lifestyles such as overeating and overwork [4]. In recent years, the treatment of acute pancreatitis is usually based on conservative medical treatment. Compared with early surgical treatment, the cure rate of patients can be increased by 70%. The main treatments include traditional Chinese medicine treatment, fasting and gastrointestinal decompression, supportive treatment, inhibition of pancreatic secretion and pancreatic enzyme activity, correction of internal environmental disorders, and maintenance of organ functions. At the onset of the disease, the patient will have clinical symptoms of gastrointestinal dysfunction such as nausea and vomiting, obvious abdominal distension, slow bowel movements, and disappearance of bowel sounds on auscultation. As one of the body's most important barriers, the intestinal barrier can effectively prevent bacteria and toxins in the intestine from entering the blood. Once dysfunction occurs, it will cause intestinal infection and endotoxemia, which will further aggravate the early acute inflammatory response, induce multiple organ dysfunction, and cause the first peak of death in acute pancreatitis. It has been confirmed that the degree of early intestinal mucosal damage in patients with acute pancreatitis is related to the severity of the disease, the total length of hospital stay, and the prognosis. Therefore, actively treating the primary disease, controlling inflammation, protecting and restoring the intestinal barrier function, and improving the intestinal microcirculation have become the key to early treatment (onset to 2 weeks).

This paper explores the effect of early enteral nutrition nursing on patients with severe acute pancreatitis and the improvement of patients' mental health and inflammation levels to provide more effective nursing methods for subsequent patients with severe acute pancreatitis.

## 2. Related Work

Due to fasting, loss of fluid in the third space, and increased vascular permeability caused by systemic inflammation, SAP patients will experience volume failure. As to whether the expansion is based on crystals or colloids, there are still differences. The guidelines for the method of fluid resuscitation are dynamic monitoring of CVP or PWCP and HCT as a guide for volume expansion and attention to the ratio of crystals to colloids to reduce fluid retention in the interstitial tissue. Xu et al. [5] believe that whether the effect of fluid resuscitation can be sustained is also affected by many factors. The first is whether the treatment to remove the cause is timely. If the cause continues, the development of pancreatitis will not be terminated; otherwise, the internal environment can only be temporarily stabilized. Secondly, it is necessary to understand the secondary changes of the disease and take corresponding treatments, such as the judgment and treatment of capillary leakage, intra-abdominal hypertension, retroperitoneal bleeding, and bowel involvement.

Abdominal pain is one of the main symptoms of SAP patients, and adequate pain control is essential for many patients. Using only acetaminophen and non-steroidal anti-inflammatory drugs often cannot solve the problem, especially when the patient has hypovolemia and oliguria, and the latter should be used with caution. Opioid analgesics are often used, but there is no research to prove which opioid is better [6]. A foreign randomized controlled trial (107 patients) showed that the effect of continuous intravenous infusion of procaine was significantly lower than that of opioids such as analgesics [7]. Piper [8] pointed out that analgesia can be considered when patients have severe pain. Under close observation of the condition, pethidine hydrochloride can be injected. Morphine or cholinergic receptor antagonists, such as atropine, 654.2, are not recommended because the former will contract Oddi's sphincter, and the latter will induce or aggravate intestinal paralysis.

SAP patients often experience organ dysfunction, and they can even progress to multiple organ failure within a few hours after the onset of clinical symptoms. According to literature [9], 56.63% of SAP patients will have respiratory failure, 23.51% will have shock, 13–42% will have renal failure, and 19–42% will have coagulation disorder, so early monitoring and treatment are very important. It is necessary to observe body temperature, pulse, respiration, blood oxygen saturation, central venous pressure, abdominal pain, and abdominal distension and pay attention to the nature, location, and degree of abdominal pain. At the same time, it is necessary to control blood sugar and closely monitor serum electrolytes, timely and effective drainage, and multi-organ support therapy. When necessary, mechanical ventilation PEEP and hemofiltration therapy are adopted. In recent years, the efficacy of traditional Chinese medicine has also been affirmed. For example, full abdominal external application of Glauber's salt, nasal feeding with rhubarb and Glauber's salt, and retention enema play a positive role in protecting organs and reducing complications.

Liu et al. [10] pointed out that SAP patients should start enteral nutrition as soon as possible because enteral nutrition can regulate the body's stress response, shorten the course of the disease, and improve the outcome of the patient. Zare Shoki and Kalhor [11] randomly divided 70 SAP patients (APACHE II score > 8 points, high CT score, and/or C-reactive protein > 150 U) into total enteral nutrition group (TEN) and total parenteral nutrition (TPN) group, and all patients were given prophylactic antibiotics. The results showed that the incidence of multiple organ failure in the TEN group was lower than that in the TPN group (20% and 50%, *P* < 0.05), the infection rate of pancreatic necrosis was lower than that in the TPN group (20% and 74%, *P* < 0.001). And the TPN group needs surgical treatment. The proportion of surgical intervention (25% and 88%, *P* < 0.001) decreased. In addition, what is more striking is that compared with previous research reports, the mortality rate of the TEN group was significantly reduced (6% and 35%, *P* < 0.001). The non-randomized study in the literature [12] also demonstrated Petrov's conclusions. The study was a 6-year prospective before-and-after controlled study with 87 SAP patients. In the first 3 years, 43 patients received TPN, and within 3 years, 44 patients received TEN. Patients who did not receive prophylactic antibiotics and those who did not receive enteral nutrition within the first week were excluded. The results showed that the incidence of multiple organ failure (57% and 85%), the infection rate of pancreatic necrosis (20% and 74%, *P* < 0.001), and the proportion of surgical intervention (25% and 88%, *P* < 0.001) in the TEN group) significantly reduced. Finally, the mortality of the TEN group was also significantly reduced (5% and 35%, *P* < 0.0001). This latest study found that enteral nutrition has become the “gold standard” of nutritional therapy for SAP patients [13]. At present, one of the main mechanisms for the effect of enteral nutrition is that enteral nutrition can increase the permeability of the intestinal wall. In addition to the nutritional approach and timing, scholars have also discussed the optimal formula of the nutrient solution. Chen et al. [14] studied the two formulas of semi-element type (using short peptide as nitrogen source) and polymeric type (using whole protein as nitrogen source). It was found that SAP patients had better tolerance to both, but the semi-element formula group had less hospital stay and lower weight loss. This shows that for SAP patients, the semi-elemental formula seems to have more advantages.

## 3. Information and Methods

### 3.1. Clinical Information

From January 2018 to December 2020, 110 patients with acute severe acute pancreatitis in a hospital were selected and grouped according to the nursing intervention plan. Observation group: 55 cases, 27 males/28 females, aged 30–72 years, mean (50.4 ± 0.4) years old. Control group: 55 cases, 29 males/26 females, aged 29–73 years old, mean (50.4 ± 0.5) years old. The basic data of the 2 groups are comparable (*P* > 0.05) [15].

### 3.2. Methods

Both groups of patients were given early enteral nutrition support. After the naso-intestinal tube was placed, the patients were provided with early enteral nutrition support. On the day of intubation, the patient was given 20–30 ml/h of normal saline for pumping. If well tolerated, the next day, the patient will transition to a short peptide preparation, 25.2 ml/h, and then the dose was increased to 80.2 ml/h within 2-3 days. After that, the dosage and low speed should be adjusted reasonably in combination with its tolerance. The patient's enteral nutrition was 104.7 kJ/kg ∗ d non-protein calories. On this basis, the control group should be given routine care, doctors should strictly follow enteral nutrition support, the speed of the nutrition pump should be adjusted reasonably, the patient's status during the infusion period should be closely monitored, and symptomatic care should be given. The observation group used comprehensive nursing intervention, and the methods were as follows. (1) Psychological nursing: on the basis of communicating with patients, it is necessary to assess their mental state and explain the relevant knowledge of enteral nutrition support and diseases to the patients in a targeted manner. At the same time, it is necessary to ensure that patients can understand the purpose and significance of early enteral nutrition support to improve patients' anxiety, worry, and other negative emotions and improve their cognitive level. In addition, it is necessary to provide targeted guidance to patients, guide family members to provide family support and care for patients, and help patients build confidence in rehabilitation. (2) Nutrient solution preparation and care: after the nutrient solution is prepared, it must be fully stirred. At the same time, it is necessary to follow the aseptic procedure during the configuration and store it in a low-temperature refrigerator. Moreover, it is necessary to ensure that the nutrient solution is prepared and used now, that is, the application must be completed within 24 hours after configuration. (3) Nutrient solution injection care: it is necessary to closely monitor the patient's reaction during the period of nutrient solution injection, reasonably adjust the infusion rate, and properly fix the patient's naso-intestinal tube to prevent pipeline deformation and distortion. Before and after the reinfusion, the pipes need to be fully flushed with warm water. At the same time, it is necessary to assist the patient in adjusting the position during the infusion and closely monitor the nutrient solution's actual dissolution. If the pipeline is blocked, it needs to be treated immediately to facilitate the pipeline to be cleared. (4) Staged care: it needs to be further divided into unstable period, disease transition period, safety period, and recovery period based on the patient's condition. Corresponding nursing interventions need to be combined with the situation of each stage. For example, in the unstable period, it is necessary to strengthen the inspection vision, monitor vital signs, and report the abnormal situation immediately. In the transitional period, psychological counseling and health knowledge education are required to improve patient compliance. In the safe period, it is necessary to ensure the patients' good medication compliance and explain the self-care methods to them to improve their self-care ability. It is necessary to give lifestyle guidance during the recovery period to enable patients to participate in sports exercises, thereby improving their physical fitness [16].

### 3.3. Evaluation Criteria

(1) The experiment uses APACHE II score to evaluate the patient's condition before and after care. (2) The experiment compares the changes of anxiety and depression before and after care of the two groups of patients, using SAS and SDS scales. (3) The experiment compares the immune function indexes of the two groups of patients before and after nursing, namely, IgG, IgM, and IgA.

### 3.4. Statistical Methods

SPSS19.0 analysis was performed on the data in the text, *t*/*χ*^2^ tested the data between groups, and *P* < 0.05 indicates statistical significance.

## 4. Results

This paper studies the efficacy of early enteral nutrition nursing for patients with severe acute pancreatitis. It analyzes the results with statistical methods, mainly evaluated from the patients' curative effect, mental health, and improvement of inflammation levels. The statistical results are shown in Tables 1–3 and Figures 1–3, respectively.

## 5. Discussion and Analysis

From the above studies, the statistical results of the efficacy of early enteral nutrition nursing for patients with acute severe acute pancreatitis can be obtained. The test results of the patient's curative effect, mental health, and the improvement of inflammation levels can be seen in the test group which are significantly higher than those of the control group, and the difference is statistically significant (*P* < 0.05) [17].

Acute severe acute pancreatitis mainly manifests symptoms such as acute abdominal pain, nausea, vomiting, fever, and increased blood pancreatic enzymes. In severe cases, pancreatic hemorrhage and necrosis may occur, complicated by infection, peritonitis, and shock, which threaten the life and health of patients. During clinical treatment and nursing, appropriate interventions to restore the barrier function of the digestive tract, regulate endocrine, and strengthen its immune function can effectively improve the prognosis. Patients with severe acute pancreatitis need necessary fasting and drinking water in the treatment process to ensure the smooth progress of the later treatment process. However, the patient is in a highly stressed state at the time of the onset, the catabolism rate is significantly increased, and the energy consumed is 2-3 times higher than that of normal people.

Moreover, the human body also needs the necessary nutrition to maintain the body's normal operation, so nutritional support is very important. The main selection of nutritional support is based on whether the patient's condition allows eating through the gastrointestinal tract, whether the gastrointestinal supply can meet the patient's needs, whether the patient's gastrointestinal function is disordered, and whether there are contraindications for parenteral nutrition support (heart failure, renal dysfunction, and so on). In the past, the most commonly used clinical nutritional support program was total parenteral nutritional support. However, clinical practice has shown that long-term uninterrupted parenteral nutrition support has certain limitations. The main manifestations are as follows: due to long-term fasting and drinking, the quality of the small intestinal mucosa will correspondingly decrease, which will damage the intestinal barrier function to a certain extent, and then the intestinal barrier function will be in an abnormal state.

Moreover, when the original barrier function is weakened, intestinal bacteria will shift in a wide range, which greatly increases the probability of concurrent infection after pancreatic necrosis and increases the mortality rate of patients. Enteral nutrition can protect patients' gastrointestinal function, enhance immunity, and accelerate gastrointestinal recovery. The reason is as follows. Enteral nutrition is the direct supplement of food into the gastrointestinal tract, and the body autonomously takes in nutrition. Compared with parenteral nutrition, it is consistent with the patient's physiological characteristics and has a more significant nutritional support effect.

Moreover, enteral nutrition support can stimulate the release of gastrointestinal hormones and has a good effect in maintaining the intestinal mucosal barrier function, thereby inhibiting the translocation of intestinal bacteria and endotoxins. Moreover, it can achieve the effects of regulating the intestinal immune response, repairing the intestinal barrier function, and maintaining the normal pH value in the stomach. After patients with acute severe acute pancreatitis are given early enteral nutrition nursing, the patients' malnutrition can be relieved and the gastrointestinal mucosal function can be protected. At the same time, it accelerates the blood circulation of the patient's internal organs, prevents the production of vasculitis, and can weaken nutrients to stimulate the intestines and stomach, shorten the duration of abdominal pain and bloating, and reduce the risk of infection. In this study, after one week of intervention, the serum albumin, hemoglobin, and plasma prealbumin of the two groups are higher than those before the intervention, and the above indicators of the test group are higher than those of the control group. After 1 week of intervention, the two groups of CD3+, CD4+, CD4+/CD8+, IgM, IgG, and IgA are all higher than those before the intervention, and the above indicators of the test group are higher than those of the control group. It shows that early enteral nutrition nursing can improve the nutritional status of patients with acute severe acute pancreatitis, enhance their immune function, and promote their disease outcome [18].

Patients with severe acute pancreatitis are usually in a state of excessively fast metabolism and consume the body's nutritional reserves quickly. When the patient is fasted with water and food, it can quickly reduce nutritional deficiencies and immunity, easily inducing various infections and damage to the gastrointestinal tract. The nutritional support makes up for the lack of nutrition in patients and the rapid decline of the body's immunity. It regulates the patient's metabolic function through nutrient solution, maintains the patient's body structure, and promotes the anabolism of the patient's body, thereby actively blocking the patient's pathological deterioration process and helping the patient's body recovery.

The medical staff provided psychological care for the patients' worries and fears due to the implementation of enteral nutrition support to help patients understand the importance of nutritional support, stabilize the patient's mood, improve the patient's treatment compatibility, and perform enteral nutrition nursing. Moreover, they use enteral nutrition support to help patients replenish body nutrition and reduce adverse effects. Before medication, the normal saline should be preheated first and then mixed and diluted to avoid adverse reactions. At the same time, it is necessary to prevent the patient from developing diarrhea due to the rapid infusion rate or the high concentration of the nutrient solution. Moreover, medical staff should pay close attention to the patient's reaction when applying nutritional support to avoid regurgitation into the stomach. After the overall nursing of patients with acute pancreatitis, the overall tolerance was good. Only two patients had mild reactions, and effective intervention was given to correct them in time. Therefore, the nutritional status of patients with severe acute pancreatitis has been effectively improved. They have all recovered and been discharged from the hospital.

In summary, when early enteral nutrition nursing is used in patients with acute severe acute pancreatitis, it has a certain effect in improving their nutritional status, regulating immune function, and promoting mental health [19].

## Figures and Tables

**Figure 1:** Statistical diagram of comparison of patients' curative effect.

**Figure 2:** Statistical diagram of comparison of mental health.

**Figure 3:** Statistical diagram of comparison of improvement in inflammation level.

**Table 1:** Comparison of patients' curative effect.

No.	Control group	Test group
1	90.2	95.7
2	84.9	97.0
3	84.3	94.5
4	89.3	92.1
5	89.6	93.2
6	84.2	96.6
7	84.8	96.6
8	88.0	95.8
9	89.3	94.7
10	90.3	96.6
11	90.9	92.0
12	90.0	92.8
13	86.5	96.0
14	85.2	95.5
15	87.8	96.5
16	86.0	92.8
17	89.2	95.8
18	84.8	94.9
19	85.8	95.5
20	88.1	96.9
21	87.6	95.7
22	89.3	93.7
23	86.8	92.7
24	87.6	95.7
25	85.5	92.6
26	88.2	96.1
27	87.2	92.5
28	89.1	94.1
29	86.6	93.6
30	85.6	94.1
31	90.4	96.4
32	88.2	93.1
33	87.5	96.5
34	90.2	96.9
35	90.2	95.5
36	88.5	94.3
37	84.2	94.9
38	84.3	92.0
39	90.9	95.8
40	90.8	93.7
41	84.9	93.8
42	87.4	94.6
43	84.1	92.4
44	89.3	92.6
45	87.8	96.5
46	85.7	94.8
47	90.0	96.9
48	87.2	93.6
49	84.8	94.2
50	90.2	92.7
51	84.2	93.6
52	88.2	93.4
53	85.9	95.2
54	90.5	93.7
55	88.3	96.8
56	84.3	97.0
57	89.3	92.7
58	89.2	93.4
59	85.8	92.5
60	84.9	94.1
61	89.3	92.6
62	86.6	94.9
63	88.6	92.6
64	87.2	93.6
65	84.8	92.3
66	85.5	95.2
67	85.2	92.1
68	85.0	95.3
69	85.1	94.3
70	84.4	94.7
71	84.8	95.0
72	90.4	94.6
73	86.6	92.3
74	88.8	93.2
75	90.9	93.6
76	86.7	95.0
77	87.9	96.5
78	85.0	92.3
79	84.5	96.7
80	90.1	93.6
81	86.6	93.8
82	86.0	95.1
83	90.6	92.5
84	89.5	94.4
85	90.1	96.7
86	88.2	93.1
87	90.4	92.4
88	88.4	93.2
89	85.1	95.9
90	85.9	95.0
91	86.3	95.8
92	85.0	96.5
93	85.9	96.8
94	89.3	92.7
95	88.6	96.0
96	87.9	93.7
97	88.5	93.9
98	88.5	93.4
99	90.1	96.2
100	84.9	92.6
101	85.9	97.0
102	84.5	94.2
103	87.5	93.7
104	89.1	93.8
105	87.3	93.7
106	84.8	96.0
107	84.9	94.9
108	89.8	93.5
109	86.5	96.7
110	85.1	93.9

**Table 2:** Comparison of mental health.

No.	Control group	Test group
1	83.7	93.6
2	91.4	92.5
3	91.9	90.3
4	81.0	86.7
5	83.0	89.9
6	85.2	90.5
7	90.1	88.6
8	89.0	91.7
9	85.3	87.1
10	84.4	86.9
11	90.7	94.6
12	88.5	94.4
13	85.8	93.3
14	87.4	87.8
15	87.1	87.8
16	82.6	86.7
17	84.0	92.3
18	85.6	92.9
19	89.7	86.1
20	86.3	89.0
21	82.3	92.9
22	87.2	90.9
23	84.6	94.4
24	84.0	92.6
25	89.2	94.7
26	82.4	92.0
27	81.9	93.4
28	82.8	94.5
29	82.9	90.3
30	88.0	90.8
31	85.5	90.7
32	86.9	88.5
33	90.9	89.5
34	86.7	90.8
35	88.4	92.2
36	90.4	92.3
37	82.5	94.8
38	86.8	93.0
39	88.0	87.6
40	90.9	91.5
41	85.6	93.9
42	87.7	91.9
43	86.3	90.8
44	85.1	88.0
45	90.1	86.6
46	90.9	90.7
47	91.9	86.8
48	83.8	93.6
49	82.2	87.8
50	87.4	89.9
51	85.5	92.2
52	83.4	92.9
53	88.1	88.0
54	89.3	92.3
55	89.9	93.5
56	84.6	90.4
57	87.6	90.4
58	90.2	87.3
59	85.3	86.6
60	89.0	92.2
61	89.0	93.8
62	81.3	94.4
63	87.2	92.6
64	82.3	93.7
65	88.4	90.7
66	86.8	89.2
67	82.8	90.9
68	89.6	94.8
69	89.1	93.6
70	88.6	90.0
71	86.0	93.9
72	88.2	90.4
73	91.7	91.7
74	85.9	87.0
75	90.4	93.6
76	84.8	86.4
77	81.1	92.0
78	83.1	92.6
79	83.6	93.9
80	86.8	92.7
81	88.9	90.3
82	82.4	91.1
83	81.9	91.4
84	85.0	90.1
85	85.7	93.3
86	82.2	88.6
87	88.9	94.8
88	85.4	94.9
89	92.0	94.8
90	82.9	94.9
91	89.0	86.5
92	89.1	89.5
93	83.1	91.0
94	88.0	88.4
95	87.8	93.2
96	83.4	91.6
97	84.8	87.1
98	82.7	88.9
99	85.2	88.0
100	82.5	94.4
101	87.2	93.6
102	88.2	93.8
103	85.4	90.7
104	91.3	90.7
105	85.1	93.4
106	91.3	86.9
107	89.9	92.4
108	83.2	89.8
109	86.1	92.2
110	84.0	91.8

**Table 3:** Comparison of improvement in inflammation level.

No.	Control group	Test group
1	93.6	95.8
2	89.2	97.7
3	89.8	92.2
4	90.3	95.4
5	88.7	97.4
6	87.8	95.4
7	87.7	96.8
8	87.7	92.6
9	91.5	96.8
10	88.8	92.5
11	87.2	95.7
12	92.0	97.7
13	89.6	97.5
14	91.0	94.1
15	90.3	94.8
16	90.1	96.9
17	92.1	98.1
18	90.2	95.0
19	88.8	93.3
20	92.7	93.2
21	89.1	93.9
22	90.9	92.4
23	92.0	98.4
24	90.6	94.1
25	92.7	98.6
26	91.0	97.4
27	89.0	95.1
28	93.2	93.7
29	91.8	97.5
30	89.7	93.5
31	89.4	98.5
32	87.9	94.2
33	89.2	94.7
34	88.9	92.4
35	92.5	96.1
36	91.5	94.0
37	87.2	96.6
38	90.2	97.8
39	90.8	98.9
40	90.2	98.6
41	87.0	95.6
42	87.6	93.0
43	87.7	97.2
44	91.2	94.6
45	88.3	92.6
46	88.0	93.8
47	87.7	98.9
48	91.7	97.1
49	88.6	97.7
50	92.9	95.6
51	89.9	93.0
52	92.8	94.0
53	92.5	96.9
54	88.1	96.0
55	90.6	95.0
56	89.2	93.6
57	88.7	96.5
58	93.2	98.1
59	92.1	96.9
60	89.2	95.0
61	92.6	97.9
62	88.6	92.6
63	93.8	95.8
64	92.6	96.0
65	92.8	98.7
66	88.8	97.6
67	92.6	94.3
68	92.1	97.6
69	88.1	94.8
70	90.1	95.7
71	91.9	97.1
72	92.6	93.7
73	87.3	93.6
74	90.7	92.3
75	92.6	98.1
76	89.3	97.8
77	90.2	92.4
78	93.2	94.3
79	92.4	92.4
80	87.1	95.4
81	93.3	95.7
82	89.7	95.4
83	87.9	97.8
84	87.0	93.5
85	90.1	96.8
86	92.0	98.6
87	89.0	97.0
88	93.2	94.5
89	87.3	93.2
90	92.7	93.2
91	88.7	98.8
92	92.7	96.8
93	93.7	98.8
94	87.5	96.3
95	93.0	95.6
96	89.7	96.0
97	89.8	96.5
98	93.9	92.1
99	89.8	98.4
100	90.2	98.8
101	90.6	96.9
102	92.3	96.0
103	92.0	95.5
104	87.0	92.2
105	90.9	93.8
106	89.2	99.0
107	90.2	95.9
108	89.2	97.7
109	93.8	97.9
110	92.2	94.8

## Data Availability

The data used to support the findings of this study are included within the article.
